# A Study of Occupational Therapy Strategies and Psychological Regulation of Students' Internet Addiction in the Mobile Social Media Environment

This article has been retracted.

**DOI:** 10.1155/2022/7598471

**Published:** 2022-09-14

**Authors:** Xueqin Zhang

**Affiliations:** School of Marxism, Zhengzhou University of Light Industry, Zhengzhou Henan 450001, China

## Abstract

This paper provides an in-depth research analysis of occupational therapy strategies and psychological regulation of students' Internet addiction in the existing mobile social media environment. Based on the definition of Internet use peer pressure, a preliminary scale with 2 dimensions of specific behavioral pressure and psychological cognitive pressure was developed. First, a professor of mental health education and a master's degree student in mental health education were invited to rate the scale, while 47 junior high school students were selected to try the scale to ensure that the questions of the scale were clearly expressed. Secondly, 461 subjects were selected to take the initial test of the scale, and item tests and exploratory factor analysis were conducted to ensure that the structure of the scale was as expected and the scale was expressed to psychometric standards. Finally, 810 subjects were selected for the scale retest, and item analysis and validated factor analysis were conducted, and their results met the psychometric criteria. Student peer attachment significantly and positively predicted adolescent Internet addiction; Internet use peer pressure played an incomplete mediating role in the prediction of peer attachment to Internet addiction; loneliness played a moderating role in the pathway of peer attachment to Internet addiction, and loneliness also played a moderating role in the pathway of peer attachment to Internet use peer pressure. The attitude towards online games is entertainment to kill time, a tool to escape the pressure of study and to gain the fun of friends comparing with each other. The main online motivations of adolescents included individual and situational factors, and behaviors were characterized by pan-entertainment and gamification, mainly through mobile social networks to obtain external information and knowledge, maintain interpersonal relationships, and gain a sense of belonging; they were characterized by a fixation on time, space, and online content. The interaction of family members is more of a behavioral habit, and the communication habits and behavior patterns established in the family will influence the construction of children's relationships with others, while parents' head-down behavior will also influence children's attention to various needs of an Internet-dependent behavior problem, which in turn affects children's problem-solving and intimate relationships with family members.

## 1. Introduction

The convenient and multifunctional services provided by social networks enable college students to interact with multiple others in multiple regions at the same time without leaving home, which reduces the cost of interpersonal communication. At the same time, online communication reduces the tension and awkwardness of face-to-face communication, especially for college students with social phobia and poor interpersonal relationship problems; the emergence of social networks makes up for their interpersonal communication needs in real life. Therefore, with the emergence of social network addiction and other related problems among college students, it is extremely important to strengthen the research on the tendency of social network addiction among college students, to distinguish those who have social network addiction tendencies, and to study their influencing factors and intervention means [1]. This will help us to adopt scientific and reasonable prevention and intervention measures to reduce the level of social network addiction among college students, guide them to use social networks scientifically and reasonably, and provide references to alleviate the negative effects of social network use on individual physical and mental development in the new media era and prevent college students from falling into the path of social network addiction. Psychosocial therapy models have been influenced by various other theories in their development, such as psychoanalytic, ego, and learning theories in psychology, role, and interaction theories in sociology, family theories, and system theories in anthropology. The emergence of social networks has accelerated the transfer of the fear of missing out from traditional offline to online contexts, and social networking media can facilitate the establishment of social connections and access to information. It is common for adolescents to learn, acquire information, exchange ideas, build relationships, and relax in the online world. However, overindulgence on the Internet can cause many problems for families and society. Some survey results show that adolescents generally have longer and earlier access to and use of the Internet despite their young biological age, making it particularly important to study adolescent Internet use.

With the popularity of the Internet and the number of network devices, increased students are getting in touch with the Internet. Because the Internet is interesting, fresh, and fast, online games, short videos, and online novels have become topics of conversation among secondary school students in their leisure time. In the context of the student Internet trend, as a secondary school student, you need to understand or use the Internet to get yourself into the Internet trend [2]. However, it is worth noting that there are still some students who do not have access to the Internet or are unwilling to actively engage with the Internet, and these students will inevitably be directly or indirectly excluded or isolated by such an Internet trend [3]. They may be under constant pressure from their peers in using the Internet, or they may spend more time on the Internet to bridge the gap between themselves and their classmates on the Internet. The former may cause adolescents to be under peer pressure to use the Internet for long periods, while the latter has a greater potential to cause adolescents to become addicted to the Internet. Both the former and the latter can be harmful to the mental health of adolescents [4].

Measurement instruments for Internet use peer stress are also not abundant and comprehensive. Through this study, a standardized and validated Internet use peer stress scale is developed to understand the status of Internet use peer stress among adolescents. There is a difference between Internet addiction and alcohol, tobacco, drug, and other substance addictions. Internet addiction does not produce physical or substance dependence, but plays a key role at the psychological level. At the same time, the causes of Internet use peer stress and the relationship between Internet use peer stress and Internet addiction are discussed, and new research directions are proposed for the theoretical construction of Internet addiction in adolescents. Some secondary schools are facing a shortage of mental health teachers, and secondary school students cannot get timely help from mental health teachers. To provide more secondary school students with timely professional psychological intervention and effectively address the psychological problems faced by secondary school students, self-help drawing therapy was developed in this study. Through the development of self-help drawing therapy themes by the counselor, others can intervene on behalf of the mental health teacher and without the professional requirements of counseling. This provides a new way of thinking for schools that lack mental health teachers, reducing the burden on mental health teachers while reaching more middle school students.

## 2. Related Works

In human interaction, you can contact any stranger with as few as six messaging sessions. In other words, you can get to know the people you want to know through only six people at most [5]. Based on this, social network-oriented Internet services were developed, i.e., social networking through “friends of friends,” which was the prototype of early social networking sites. Mahapatra defined social network addiction as an individual's excessive use of social networks despite their negative effects on social activities, learning, work, relationships, and mental health [6]. Social network addiction is a tendency for individuals to compulsively use social networks despite the negative consequences, to be emotionally involved in social networks, and to have negative emotions when they are restricted or unable to use social networks [7]. It is also clear from the concept of fear of missing out that individuals who fear missing out are concerned about missing meaningful experiences of others and that individuals who continuously participate in social activities or check social media are the external behavioral manifestations of the fear of missing out, while strong expectations of knowing what others are doing are the internal cognitive manifestations of the fear of missing out [8]. As a subtype of anxiety, individuals who experience fear of missing out are bound to seek specific channels or platforms to reduce their anxiety levels, and social networks are a convenient and quick channel to reduce fear of missing out [9].

Internet dependence is different from Internet addiction [10]. The dependent person does not have addictive substances and does not show withdrawal symptoms and strong psychological craving for addictive sources like an addict, but only a mild mental addiction and habitual Internet behavior [11]. He must understand his environment and the state of interaction between his family, school, friends, and other social groups. They see the Internet as a safe place where they can find solace and identity, relief, and stimulation. When encountering frustration and difficulties, the dependent person tends to retreat to what he considers a safe and familiar online world [12]. Therefore, the psychological study of Internet-dependent groups is also an important aspect of Internet addiction research and an important element to be explored. Based on the compensation model, the use of the Internet alleviates real-life psychological problems as well as unmet needs, and individuals may have a stronger desire to spend more time online, but excessive use can lead to problematic outcomes, i.e., Internet addiction [13]. With the ubiquity of the Internet in society, it is even more important to understand the context, purpose, and motivation of Internet use in this context, and some of the symptoms of addiction can be interpreted as a shift in the norms of entertainment or communication in the younger generation and show the embeddedness of the Internet in everyday life rather than pathological behavior [14].

The degree to which a person is separated or connected to his or her family system and the degree to which family members subjectively experience mutual emotional connection, including consistency in proximity, time and space spent together, and chatting styles among members are referred to as family closeness. The degree of flexibility and resilience of the family system to deal with problems is the focus of family adaptability and is defined as the ability of the marriage or family system to change in response to problems in different stages of development, the adjustment of role orientation and sociability rules, focusing on the ability to change family situations. When family members change, especially when family members change their expectations, individuals and family systems are in a constant state of flux as the family develops over time and the dynamics of the family environment evolve, with changes in closeness and adaptability. From the formation of a family to the birth of a child to school to adolescence to the beginning of independence in the face of society, these things change to reflect the stability of the family system and the growth needs of family members, and changes in the relationship between parents and children reflect the behavior patterns in the family system, for example, in adolescence when the two tendencies of attachment to parents and self-awareness of independence temporarily enter a stage of conflict and confrontation.

## 3. Analysis of Occupational Therapy Strategies and Psychological Regulation of Students' Internet Addiction in the Mobile Social Media Environment

### 3.1. Occupational Therapy Strategies for Students' Internet Addiction in the Mobile Social Media Environment

Friends usually play the exact opposite role of parents when it comes to Internet use. As parents, they usually try to limit their teenagers' excessive Internet use [15]. However, the excitement generated by the virtual world only exists when teenagers enter the bizarre online world and bizarre online games. Conversely, peers may prolong Internet use because Internet use fosters relationships with each other and increases the amount of common ground between them. Since the beginning when the concept of Internet addiction was accepted by some scholars and measurable programs were studied, many scholars began to investigate the relationship between peer attachment and Internet addiction. However, the conflicting results of the existing studies by many researchers on the relationship between peer attachment and Internet addiction are not only reflected in the different correlation coefficients between the variables but also reflected in the controversial direction. Empirical studies on adolescent addictive behaviors suggest that both the presence and absence of peer attitudes toward appropriate behaviors and the quality of peer relationships are important influences and predictor variables of adolescent substance addictive behaviors. However, there is a difference between Internet addiction and substance addiction such as alcohol, tobacco, and drugs, in that Internet addiction does not create dependence on a physical or material level, but plays a critical role on a psychological level. Therefore, the relationship between peer attachment and Internet addiction needs to be confirmed by further research.

The real-life environment in which adolescents live includes the surrounding world, the interpersonal world, and the world of the self, as mentioned by Rome. The interpersonal world is the specific behaviors that adolescents make in the process of socializing with the group, and their behaviors are closely related to their environment. The self-world is the self-judgment that adolescents themselves make after producing behaviors in their environment, and in this way, they position themselves in the group. As Lolomé emphasizes, loneliness arises from the positioning of oneself about others, on the one hand, and from an overemphasis on being socially accepted, on the other. This may also explain more clearly why students in a state of loneliness are willing to gain the approval of others by using the Internet more diligently. The attitude towards online games is that they are a time-wasting entertainment, a tool to escape from the stress of studying, and a way to have fun comparing friends with each other. Since the concept of Internet addiction was accepted by some scholars and developed a measurable solution, many scholars began to study the relationship between peer attachment and Internet addiction. They are indifferent to issues concerning their parents, resist them, and often complain about their parents' lack of understanding.

All subjects were divided into four groups according to the SDS scoring rules: normal depression group, mild depression group, moderate depression group, and severe depression group [16]. In essence, there is no difference from other entertainment activities, if a lot of energy and time is spent on Internet entertainment, it will affect normal study, work, and even physical and mental health, the formation of Internet addiction means that people spend a lot of time and frequency of entertainment on the Internet beyond their previous plans and expectations, and they cannot control it effectively from the subjective point of view, and after taking coercive measures, they produce a series of maladaptive symptoms, resulting in the behavior that cannot effectively control the frequency and time of Internet access, as shown in Table 1.

Both were busy managing the store most of the time and because they lived above the store, the boundaries between work and life were not clear and time could not be completely separated. Both parents blurred the boundaries between work and life and often spent the time they would have spent together as family members tending to the store. Once they leave their mobile phones and the Internet, the most obvious emotions when they are trapped in the virtual network begin to show. For example, when the family is eating and talking upstairs, they must go downstairs to receive customers as soon as they arrive at the store downstairs. When there is no business free, the father is often in the store playing with the computer while taking care of the merchandise, and the mother will go out to shop with friends after finishing the household chores; while playing with the phone upstairs, the three of them do not disturb each other. The parents communicate most about whether there is enough pocket money, whether homework is completed on time, and whether there is no concern for psychological needs.

Compared to other theoretical analyses of case social work, the most distinctive feature of the psychosocial treatment model is its openness and holistic nature, which incorporates a variety of theories. Thus, the psychosocial treatment model has been influenced by various theories in its development, such as psychoanalytic theory, self-psychology and learning theory in psychology, role theory and interaction theory in sociology, family theory, and systems theory in anthropology. The psychosocial treatment model brings together these different theories to form its unique theoretical model of analysis [17]. The core of its theoretical assumptions includes the assumption of human growth, which believes that the development of an individual is influenced by three factors: physical, psychological, and social, and that these three factors interact with each other to influence the growth process of the client and the assumption of the client's problems.

In this study, the emergence of the individual client's problem is not the single cause of the client's Internet addiction problem; the influence of multiple physiological, psychological, and social factors may lead to the emergence of the youth's Internet addiction problem, so the view of the problem should not be limited to a single factor. The case service should involve the individual life, study, family, and community of the client, respectively, and fully consider the current situation of the client in specific scenarios. During the service process, not only should the client's problems be solved, but also attention should be paid to harmonizing the relationship between the person and the environment, obtaining support from the family, school, and community, and helping the client return to a normal life. Specifically, the model emphasizes a systems approach to analyzing human behavior in situations, arguing that a person is seen as a completely independent and self-existing individual and that to study a person, one must understand his environment, i.e., the state of interaction between his family, school, friends, and other social groups. The interaction between the person and the environment is of paramount importance. At this time, the client is no longer cumbersome and appears to be flexible and mobile, and the whole person is radiant; at the end of the case, the author suggested that the client should maintain the amount of exercise once a week and can take the initiative to find classmates to play with in the school physical education class. In the system of interaction between the person and the environment, changes in any part will cause changes in other parts, constantly interacting and molding each other. Therefore, it is necessary to enhance the self-adaptive capacity of the client, the function of the “human-in-context” system, and finally achieve a state of balance.

Communication theory is mainly applied to the dialogue between social workers and clients. The focus is on the control of the relationship between the two sides; i.e., social workers need to keep an active atmosphere throughout the whole practice process, prevent the case owner from withdrawing in the middle of the process, enhance the sense of participation of the service users, advocate the autonomy of the service users, and establish a social worker-case owner relationship of mutual respect and understanding [18]. An equal and harmonious communication relationship is more likely to guide the clients to form a correct outlook on life and values, rationally distinguish right from wrong, and prevent themselves from falling into various undesirable temptations.

Once people are caught in the online world, their thinking logic and rational emotions are difficult to maintain at a normal level, sometimes hyperactive, sometimes irritable, and sometimes sad, but the pleasant exhilaration generated by the virtual world only exists when adolescents enter the bizarre online world and strange online games, once they leave the cell phone and the Internet, the most obvious emotions when they are caught in the virtual network begin to show up: anxiety, boredom, and depression. It is difficult to control their temper.

At this point, the social worker then looked for volunteers in the volunteer group who could teach sports to follow up and help Peng try more sports [19]. During the subsequent sports, the client learned a new sport each time, and the one that impressed him most was volleyball. With the help of the social worker and volunteers, the client was able to dribble and catch a simple volleyball, and his arm strength was increasing. In addition, the social worker also helped him to search for a small partner in the venue who could play sports with the client for a long time so that he could also urge and motivate the client to exercise after the service was over. Before closing the case, the author, the social work team, volunteers, and the client and his partner played a friendly volleyball game. Individuals with depressive disorder have a certain degree of insight. In terms of improving the client's physical fitness and repairing damaged functions, the author chose the most direct physical exercise to help the client divert his attention and accelerate his withdrawal from Internet addiction.

### 3.2. Psychological Adjustment Analysis

Through the analysis of the data, it has been learned that among the 10 different types of school consumption, canteen consumption, supermarket consumption, and Internet consumption account for most of the total consumption, but the nature of consumption of these three consumption types is very different. Canteen consumption is the basic consumption of students, supermarket consumption represents more aspects of life and entertainment, and Internet consumption, moreover, can directly reflect the amount of time students spend on the Internet. Canteen consumption and supermarket consumption may reflect some family's economic situation, which can also indirectly reflect the influence of family's economic situation on students' Internet addiction [20]. For example, students from economically disadvantaged families may study harder and spend most of their time on study, so they may spend less time on the Internet in comparison and thus have less risk of Internet addiction. Students who are at high risk of Internet addiction may spend more money on the Internet than students who are at low risk of Internet addiction. The amount of electricity may also affect Internet addiction, and people who are at high risk for Internet addiction may use more electricity. In this section, we analyze different types of consumption, hoping to get the consumption characteristics of students with a high risk of Internet addiction and students with a low risk of Internet addiction, to provide a theoretical basis for the subsequent model prediction and thus improve the accuracy of the model.

The difference between the moderately depressed and normal groups was statistically significant, with significantly fewer subjects in the normal group choosing to use the music player-type app last before bedtime than in the moderately depressed group, but there was no statistically significant difference in the results of the normal group compared to the mildly depressed group [21]. Therefore, it may be since subjects with moderate depression have more needs to relieve negative emotions than subjects with mild depression. The music therapy in question can improve depression and sleep disorders. In general, individuals with depressive disorders have a certain level of self-awareness, so subjects with moderate depression may have a greater need to relieve negative emotions than those with mild depression and choose to play music at bedtime to improve their mood problems and sleep quality, while those with mild depression have a less urgent need than those in the moderately depressed group and therefore have a lower need than those in the SDS group. Mildly depressed individuals had fewer pressing needs than moderately depressed individuals and therefore did not show statistical differences from the normal group.

In the double-choice question on the location of most frequent smartphone use, there was a significant difference between the normal and mildly depressed groups of depression scores. The percentage of the normal group and the mildly depressed group who chose to use their smartphones most often while on the road was 12.10% and 20.40%, respectively. The percentage of subjects who chose to use their smartphones most often while studying or working was only 6.50% in the normal group, but up to 15.6% in the moderately depressed group, with a statistically significant difference. This study developed a self-help painting therapy. With the counselor developing the topic of self-help drawing therapy, others can intervene on behalf of the mental health teacher and there is no professional requirement in counseling. The use of smartphones while studying or working is a safety risk, and subjects who choose to use their phones most often while on the road may have less self-control and more dependence on their phones. Self-control refers to the process by which individuals consciously control their behavior and try to change their responses to external stimuli, rather than trying to change the external environment. According to the dual system model theory, self-control is defined as the impulse system and the self-control system. People who score high on the impulse system react more directly and quickly but have a lower ability to resist temptation, while those who score high on the self-control system think and plan before reacting to specific events and are more resistant to temptation.

The results of the ANOVA of college students' propensity to social network addiction and their scores on each dimension at their fathers' literacy level showed that the main effect of literacy level was not significant, as shown in Figure 1.

If the total effect is significant, the mediating effect stance is used, and if not, the masking effect stance is used [22]. The model fitting results showed that the total effect of family closeness and adaptability on network dependence was significant, indicating that this study can stand on the mediating effect and proceed to the next step of the analysis. The emergence of social networks has compensated for their need for interpersonal communication in real life. The standardized path coefficient of family closeness and adaptability on network dependence was 0.26, indicating that family closeness and adaptability can negatively predict network dependence; i.e., the higher the individual's family closeness and adaptability, the lower his or her network dependence is. The findings suggest that the path coefficient is significant and allows for subsequent mediating effects.

The overall level of Internet dependence is moderately low, among which the detection rate of pathological Internet use group is 6.7%, the detection rate of marginal Internet use group is 3.3%, and the detection rate of normal Internet use group is 90%. The reason may be that the circular issued by the Ministry of Education to restrict the use of cell phones by teenagers at school has restricted the use of cell phones by teenagers at school to a certain extent [23]. It is obvious that both the former and the latter are harmful to the mental health of adolescents. It has become a part of their life, an auxiliary tool for learning, a platform for discussing problems, sharing experiences, exchanging opinions, and expressing views, and the first choice for leisure and entertainment.

## 4. Analysis of Results

### 4.1. Occupational Therapy Outcomes for Students with Internet Addiction

Based on the results of the meta-analysis between peer attachment and Internet addiction, Internet use behavior significantly moderated the relationship between the two. Therefore, it is necessary to conduct a difference-in-difference test based on the classification of Internet use behaviors to investigate the differences between individuals under different Internet use behaviors in each variable.

Independent sample *t*-tests were conducted on the levels of peer attachment, Internet use peer pressure, loneliness, and Internet addiction for students who did or did not play games online. The results showed that there were significant differences in the peer attachment and Internet addiction variables, with students who did not play online having significantly higher levels of peer attachment than those who played online and students who did not play online having significantly lower levels of Internet addiction than those who play online. The results of the effect sizes were found to be small for the peer attachment variable and large for the Internet addiction variable, as shown in Table 2.

Independent sample *t*-tests were conducted on the levels of peer attachment, Internet use peer pressure, loneliness, and Internet addiction for students who listened to music online or not. The results showed that there were significant differences in the loneliness variables, and students who did not listen to music online had significantly higher levels of loneliness than those who listened to music online. The results of the effect size calculation revealed that there was a small effect size for whether to listen to music online under the loneliness variable.

First, the independent and moderating variables were centered to avoid effects due to their differences or large differences in values. Second, the interaction term between peer attachment and loneliness needs to be calculated. Using validated factor analysis, the loadings of each dimension of the two variables, peer attachment, and loneliness, were calculated and ranked in a descending order of the magnitude of the dimensional loadings. Then, the interaction terms were obtained by calculating the centralized products of the factors in the order of the factor loadings following the principle of “large matches large, small matches small.” Therefore, with the continuous emergence of social network addiction and other related problems of college students today, it is necessary to strengthen the related research on college students' social network addiction tendency. Finally, by constructing a structural equation model, we investigated whether the interaction terms of peer attachment and loneliness were significant on the path coefficients of peer pressure to use the Internet and whether the interaction terms of peer attachment and loneliness were significant on the path coefficients of Internet addiction.

The moderating role of loneliness in the pathway of peer attachment to Internet use peer pressure was further explored by the simple slope. Adolescents' loneliness levels were divided into 3 groups by *M* ± 1SD, with those scoring 1 standard deviation above the mean as the high group, those scoring 1 standard deviation above the mean as the medium group, and those scoring 1 standard deviation below the mean as the low group. To test the moderating effect, the path coefficients were tested by Bootstrap 5000 times with a 95% confidence interval, and the path coefficients were tested by the great likelihood method. In the high loneliness group, the level of peer attachment significantly predicted the level of network use peer pressure (*β* = 0.28) with a 95% confidence interval of [0.13, 0.45] for the percentile Bootstrap method. 95% confidence interval was [0.20, 0.01]; in the low loneliness level group, peer attachment level did not significantly predict the level of Internet use peer pressure among adolescents (*β* = 0.11), with a 95% confidence interval of [-0.01, 0.23] for the percentile Bootstrap method. The data results indicated that peer attachment level significantly predicted the level of adolescents' Internet use peer stress in the case of high and moderate loneliness and that peer attachment level did not significantly predict the level of adolescents' Internet use peer stress in the case of low loneliness, as shown in Figure 2.

From the process of treatment and the effect of the treatment, the intervention of this case is effective to some extent. Although the client did not completely disconnect from the Internet, he had some rational knowledge about the use of the Internet and gained some obvious results: the frequency and length of time he spent on the Internet were significantly reduced; the content of the Internet was expanded from a single online game to watching movies and searching for study materials, and he had a new understanding of the correct use of the Internet; his motivation and academic performance were also improved, and the progress in single subject grades was more obvious; he got along with his family more and more and started to open up with them, and the parent-child relationship gradually developed positively. Social networking and access to information can be facilitated through social networking media. Most importantly, her self-esteem has improved, her self-efficacy has gradually increased, and she has gained confidence in her future.

The personal narratives that we often find facilitated in a therapeutic dialogue that differ from social norms are not meant to challenge these rights relationships, but rather to focus on the values and passions for life that this exceptional personal narrative reflects, creating a sense of solidarity with others, where the original story development that did not meet expectations may be less and less, but persists in such a context. Mike White refers to the outsider witnessing session as a defining ritual and distinguishes it into three stages: storytelling, retelling, and retelling. In the process of talking with the outsider witness, the focus is on understanding four types of exploration: expression, imagery, personal empathy, and transference. Imagery refers to the imagery that the case narrative evokes and how it reflects the case's goals, values, beliefs, hopes, passions, commitments, etc. These four types of explorations are very influential in enhancing the plurality of the case story, illuminating the exceptional events of the case, and enriching the branching life stories of the case.

### 4.2. Psychological Adjustment Results

Personality development reflection in the psychosocial treatment model can help clients to reacquaint themselves, review their past behaviors, adjust their personality in time, and return to normal life as soon as possible. Social workers create a more relaxed environment to stimulate Pengpeng's interest in learning by chatting and sharing interesting stories about their respective schools and studies. Through techniques such as respect and empathy, Pengpeng felt understood and supported by the social worker. Because Pengpeng is introverted and not very good at expressing himself, the social workers and volunteers actively guided him to feel every progress he made in his studies to enhance his motivation and develop good study habits. Pengpeng said he was interested in physics, so the volunteers and social workers started with physics, agreeing to write one hour of summer homework every day, mark the ones they do not know first, and then answer them after the social workers and volunteers came to the house. In addition, clients can also use the Internet to study and then search for free middle school courses or enroll in classes online. Among the donated materials received by the social work organization was a study card of HJN, which was still valid, so the social worker gave it to the client.

Understanding his love for photography, the social worker took him to the park to learn basic shooting techniques and field experiments to regulate his mood and increase his motivation to learn. In addition, the social worker worked with the classroom teacher to help Pengpeng regain his inner drive to learn. Through the help of teachers and volunteers in charge, Pengpeng was able to regain the joy of learning. Among the students in the 4 : 30 classroom, one or more sports partners are found to burn the soul of sports and enrich their spiritual world. Through the experience of nonaddicted peers, social workers guide the clients to understand and use the Internet comprehensively and correctly and use the positive influence of peer groups to encourage them to learn from each other, support each other, and supervise each other, to achieve the goal of leaving the Internet addiction. It has become very common for teenagers to acquire knowledge, obtain information, exchange ideas, build relationships, and have fun in the online world. The social worker encourages Pengpeng to take the help of the class help group seriously, learn to observe or ask for advice on the learning styles of students with good grades, and then combine them with his situation to organize his learning methods and develop his inner potential.

Based on Study 1, this study conducted six sessions of positive cognitive group counseling to improve the level of loneliness and cell phone dependence of junior high school students, which effectively enabled the participants to experience warmth and strength in the group and to become aware of their bodies and feelings, thus improving the dependence of junior high school students on cell phones. The former may cause adolescents to be under peer pressure for Internet use for a long time, while the latter is more likely to cause adolescents to be addicted to the Internet. The purpose of positive cognitive therapy is to make the participants spontaneously perceive others and the environment from within through the repeated practice of the positive cognitive technique and then return to their hearts to answer their doubts, as shown in Figure 3.

In the intervention group, there were significant differences between the pre- and posttests in the total scores of loneliness and cell phone dependence, while there were no significant differences in the pre- and posttests of the control group. The level of loneliness and cell phone dependence were significantly improved after the positive cognitive group support intervention.

The data collected were subjected to structural equation modeling, and the results of the runs were compiled and analyzed. The coefficient of the standard path effect of misinformation fear on obsessive-compulsive thinking was 0.282, which reached the significance level (*p* < 0.001), indicating a significant positive effect of misinformation fear on obsessive-compulsive thinking; the coefficient of the standard path effect of misinformation fear on mood change was 0.397, which reached the coefficient of the standard path effect of misinformation fear on social adjustment which was 0.422, which reached the level of significance (*p* < 0.001), indicating a significant positive effect of misinformation fear on social adjustment; the coefficient of the standard path effect of misinformation fear on compulsive thinking was 0.287, which reached the level of significance (*p* < 0.001), indicating a significant positive effect of misinformation fear on compulsive thinking.

The coefficient of the standard path effect of misinformation fear on compulsive thinking was 0.287, which reached the significance level (*p* < 0.001), indicating that misinformation fear had a significant positive effect on compulsive thinking. Online games, short videos, and online novels have become topics that middle school students talk about in their spare time. The coefficient of the standardized pathway for the effect of fear of missing scenarios on social adjustment was 0.225, which reached the significance level (*p* < 0.001), indicating that fear of missing scenarios had a significant positive effect on social adjustment, as shown in Table 3.

The compulsive thinking dimension of college students is higher than the total mean score of social network addiction tendency, and the mood change and social adaptability dimensions are lower than the total mean score of social network addiction tendency. Most of the students use social networks for 2-4 hours, accounting for 41.8%; there are significant differences in the tendency of social network addiction among college students in terms of gender, whether they are only students, professional category, and grade level and whether they are student leaders; there are significant differences in the social adaptability dimension among college students in terms of their mothers' cultural level; there are significant differences in the compulsive thinking dimension scores among college students in terms of whether they are in love. The above findings are both like and different from previous studies, which may be related to the differences in the geographic location, type of institution, social development in the era in which the surveyed groups are located, and the distribution of demographic variables.

## 5. Conclusion

This study developed a moderated mediation model to examine the mediating role of cell phone dependence in the relationship between Big Five personality traits and mental health and whether this role was moderated by motivation for cell phone use. It was found that in the era of mobile media, different personality traits can have both direct effects on mental health and indirect effects on mental health through cell phone dependence and that this mediating effect is also moderated by the motivation for cell phone use, which varies in intensity and has large and small mediating effects. Under the background of the trend of student Internet, as a middle school student, you need to understand or use the Internet to integrate yourself into the Internet trend. For diagnosed Internet addicts, medical personnel should carry out effective psychotherapy and necessary medical treatment and do a good job of related health education. Patients with stable symptoms of Internet addiction can be referred to community medical institutions through two-way referral, and the community medical institutions should designate a person or team to be responsible for follow-up correction and management follow-up. Community medical institutions should establish health files for diagnosed Internet addicts, sign “family doctor service agreements” if necessary, carry out regular follow-up work and health education according to the patient's condition, and communicate closely with the patient's family to regulate his or her Internet behavior. Community medical institutions can organize regular educational lectures on healthy Internet access and prevention of Internet addiction or activities on the dangers of Internet addiction with street offices or community service centers. The social treatment model allows clients to face their problems squarely by transforming their perceptions, understanding the root causes of the problems, and guiding them to build strong self-control, form correct perceptions, establish correct outlooks on life and values, and independently solve their life and study dilemmas and resist undesirable temptations even after the case is closed.

## Figures and Tables

**Figure 1:** Model of the total effect of family closeness and adaptability on network dependence.

**Figure 2:** Score measured before and after treatment.

**Figure 3:** Analysis of the overall goodness-of-fit of the model.

**Table 1:** Descriptive statistics.

Variable	*N*	*M*	*S*	SD
Understanding social support	40	43	16	50
Family support	25	37	14	29
Friend's support	32	40	53	38
Other support	19	47	13	60
Loneliness	34	56	51	60
Cell phone dependence	44	39	11	41
Out of control	50	60	13	18
Withdrawal	31	10	11	57
Escape	53	46	43	23
Inefficiency	10	30	49	46

**Table 2:** Analysis of variability in playing games online on each variable.

Variable	Whether to play games online	*t*	Cohen's *d*
Peer attachment	Yes	0.868577154	0.844699964
Internet use peer pressure	No	0.980331986	0.591271836
Loneliness	Yes	0.009234343	0.769672889
Addicted to internet	No	0.974402719	0.453188186

**Table 3:** Intermediary model with moderation.

Step	Dependent variable	Standard coefficient	Standard error
1	Mental health	Openness	3.3
2		Mobile phone use motivation	3.7
3		Openness∗ to machine motivation	5.3
4	Cell phone dependence	Openness	4.3
5		Motivation for getting off the plane	2.8
6		Independent variable	1.9

## Data Availability

The data used to support the findings of this study are available from the corresponding author upon request.
